# Urban transportation system toughness assessment under New Crown epidemics

**DOI:** 10.1371/journal.pone.0300652

**Published:** 2024-03-25

**Authors:** Tianjun Feng, Xubin Zeng

**Affiliations:** School of Transportation Science and Engineering, Jilin Jianzhu University, Changchun, Jilin, China; Zhejiang University of Technology, CHINA

## Abstract

Since the concept of toughness was introduced to transportation systems, transportation system toughness has received extensive attention from researchers in the field of transportation worldwide. In this paper, a methodology for quantifying and assessing the toughness of urban transportation systems is proposed in the context of the New Crown epidemic. Firstly, the definition of urban transportation system toughness in this context is clarified, and the entropy evaluation method is applied to construct the performance curve of urban transportation systems over time. Then, it is proposed to quantify the system’s resistance, recovery, and adaptive ability in terms of the change in the cumulative amount of system performance. Finally, the three characteristic abilities of system toughness are organically combined to obtain a comprehensive assessment of system toughness. Example calculations and analyses are carried out in four Chinese cities with different levels of development, and the results show that the performance of urban transportation systems is positively correlated with their levels of development, and all of them fluctuate greatly under the influence of the epidemic, but Wuhan has the strongest resistance and recovery ability of the transportation system, and shows the highest toughness, followed by Lanzhou, Changchun, and Shanghai. The system toughness quantification and assessment methods proposed in this paper provide a reference for research on improving the ability of urban transportation systems to deal with multiple uncertainty disturbances.

## 1 Introduction

In the context of global climate change and frequent emergencies, sustainable development is the theme of the times [1, 2], and the concept of toughness provides a new research perspective [3], which is being increasingly applied to the study of sustainable development of urban transportation systems [4] and has received extensive attention from scholars in various fields around the world [5, 6]. For emergencies such as the New Crown Epidemic, urban transportation, as a core infrastructure system for urban functioning, is a key node for maintaining commuting and rapid recovery from the epidemic [7]. However, in this context, there is less research content related to the toughness of urban transportation systems, and there exists a great deal of space for quantitative research on its toughness. When facing the new crown epidemic event, the urban transportation system [8, 9] is unprecedentedly affected [10, 11], how to combine qualitative and quantitative analysis of its system toughness, analyze the anti-interference ability, recovery ability and other characteristics of it, has become an important issue in the field of global transportation system toughness research.

Toughness is originally derived from the Latin word resilio, meaning “to reset to the original state”, which gradually evolved into the modern English word “resile”. In the 1970s, ecologist Holling [12] first described the phenomenon of multiple equilibrium states of natural systems and used the term toughness to characterize the ability of the system to absorb the impact of various types of unexpected events. Toughness is a kind of “adaptive” and “recovery” ability, its meaning can be in the uncertain conditions of the ability to adapt and recover, can also be the ability to repair the system by the external disturbance of the damage caused by the system, but also includes the system’s development ability. Based on the development of toughness theory, Murray-Tuite et al. [13] first proposed the concept of transportation system toughness and summarized 10 dimensions such as rapid recovery ability, which set off a boom in related research and practice [14, 15]. With the deepening and systematization of toughness research, the connotation of toughness has experienced from engineering toughness emphasizing “single equilibrium state” to ecological toughness emphasizing “multiple equilibrium states” to “not pursuing equilibrium state”. “Evolutionary toughness, in which the connotation of transportation system toughness [16, 17] and research [18, 19] are also constantly expanding and improving. This paper proposes that in the face of the new crown epidemic public health emergencies, the urban transportation system toughness refers to the urban transportation system in the face of epidemic interference, maintaining and restoring the normal level of service, and face the next interference, that is, the organic combination of resistance, recovery and adaptive ability.

Currently, there are several transportation system toughness assessment methods: indicator system method, Bayesian network, simulation method, and system performance curve. The assessment method based on the indicator system can highlight the toughness influencing factors, but it cannot describe the continuous change process and the dynamic balance of the system in the disturbance event. For example, Fang Dongping et al. [20] proposed the resistance to disaster and post-disaster recovery ability of urban transportation system toughness under the framework of “physical-social-informational three-degree space”, but did not consider the adaptive ability. Ji K et al. [21] constructed a safety toughness assessment index for urban rail transit from the three dimensions of adaptive, responsive, and recovery. Chen Y et al. [22] analyzed the toughness of multimodal urban transportation networks using complex network theory based on topological index. and Ma D et al. [23, 24] to improve network throughput and ensure network stability, as well as traffic flow prediction methods were inspired. Bayesian network model [25, 26] can consider many factors [15], for example, Jiang W et al. [27] mixed Bayesian network and principal component analysis to analyze China’s transportation system, but the probability of the problem of subjectivity is too large. Bai F et al. [28] used the Monte Carlo simulation method to stochastically simulate the subway network from the travel time, the number of interchanges, the node degree, the average node intermediary, and other metrics to assess the toughness of the metro network, considering only one mode of transportation. Datola G et al. [29] system dynamics modeling to analyze and simulate related urban toughness problems. The assessment method of system performance curves can consistently describe the system performance and thus characterize the change process of system toughness. For example, Wang et al. [30] assessed urban transportation toughness hierarchically, but the toughness curve fitting was too idealized, while Chen Changkun et al. [31] considered service rate and online rate to characterize the system performance. Current research such as network simulation by Kong X et al. [32], and interference research results by Zong F et al. [33] have enriched the means of toughness assessment [34], but the existing transportation toughness assessment research objects are mostly infrastructures [35] and analog simulation [36], and there are fewer researches on the system toughness assessment methods for the system containing multiple types of infrastructures and under the new crown epidemics. while less research has been conducted on the system toughness assessment methods for systems containing multiple types of infrastructures and new crown epidemics. The urban transportation system contains multiple types of infrastructures such as highways, rail lines, and other information changes such as urban passenger traffic [37], which puts forward higher requirements for toughness assessment methods.

The impact of the new crown epidemic on the urban transportation system is more in the form of disturbed system performance, which causes frequent fluctuations in performance, rather than in the form of disasters such as earthquakes, typhoons, and floods, which cause damage to the urban transportation system, or even paralyze the transportation. Therefore, in the subsequent research, the performance of the urban transportation system should be based on the urban transportation system performance, in order to make a more scientific and comprehensive assessment of the urban transportation system toughness in the context of the epidemic. Therefore, this paper proposes to construct a quantitative assessment model of urban transportation system toughness based on the system performance curve on the basis that urban transportation system toughness in the context of new crown epidemic contains three major characteristic capabilities: resistance, recovery and adaptation. In detail, it is proposed that the entropy value method is used to construct the urban transportation system performance curve, and then the mathematical integration method is used to quantitatively calculate the ratio of the cumulative amount of the system performance to the three major characteristic capabilities, which is combined to arrive at the value of the system toughness. The proposed model is applied to the transportation system of Shanghai, Wuhan, and other central cities in China as an example to provide a reference for the construction of urban transportation system toughness.

## 2 Urban transportation system toughness assessment model

This paper avoids the influence of subjective ideas of the mainstream index system method for assessment, and more objectively and scientifically assesses the urban transportation system toughness comprehensively from the three dimensions of resistance ability, recovery ability, and adaptive ability. In the face of the new crown epidemic, the entropy evaluation method is used to construct the performance curve of the urban transportation system. Then the quantitative calculation method of the urban transportation system’s toughness is proposed to achieve a comprehensive assessment of the system’s toughness.

### 2.1 Urban transportation system performance curve

#### 2.1.1 Urban transportation system performance curve concept

After facing the impact of a new crown epidemic, the urban transportation system will be shifted from the equilibrium homeostasis and undergo the dynamic process of resistance, recovery, and adaptation, as shown in Fig 1. In the figure: *Q*(*t*) denotes the curve function of urban transportation system performance over time, and *t*_0_ to *t*_4_ is the whole cycle of resistance-recovery-adaptation after the system is disturbed by the epidemic. Where: *t*_0_ represents the starting time when the system is affected by the disturbance; *t*_1_ represents the time when the system performance drops to the lowest value *Q*(*t*_1_); *t*_2_ represents the time when the system performance recovers to a certain level and no longer grows at a high speed in a short period, and tends to be stabilized or declines again; *t*_3_ represents the time when the input of materials and manpower related to the recovery of the system performance stops, which means that no more traffic under epidemic control; *t*_4_ is the cutoff time of the study.

**Fig 1:** Urban transportation system performance.

Specifically, when *t* < *t*_0_, the urban transportation system operates normally without the disruption of the new crown epidemic and the performance is maintained above and below 100%.

When *t*_0_ < *t* < *t*_1_, the system is in the resistance phase, and the system performance continues to decline due to the epidemic interference, and the lost performance of the system can be expressed by *Q*_*L*_ = *Q*_0_ − *Q*(*t*_1_). It can be seen that resistance ability means that a system with toughness can absorb the negative effects generated by the disturbance and its core functions will not be completely destroyed.

When *t*_1_ < *t* < *t*_2_, the system is in the recovery phase, and with the input of human and material resources under the policies such as control, the system function starts to recover and recover to the maximum value in the cycle, and the duration is related to the organizational capacity and resource input. To characterize the speed of system performance recovery, the average recovery rate of the system function can be measured by *v* = [*Q*(*t*_2_) − *Q*(*t*_1_)]/[(*t*_2_ − *t*_1_)]. Recover ability can be seen to refer to the measures that can be taken by the system to make it operate at the desired level after a disturbance occurs.

When *t*_2_ < *t* < *t*_3_, the system is in a situation where it is once again faced with a new crown epidemic disturbance, and the maintenance of system performance within this phase is related to the organization’s investment of human and material resources, so the level of system performance in the face of this disturbance may decline or stabilize at a certain level.

When *t*_3_ < *t* < *t*_4_, it is declared that there will be no more policy control of the new crown outbreak and the society is in a state of complete liberalization. At this time, the system is in the adaptation phase, and no more human and material resources are organized to be invested during this phase, and the system performance is free to recover. It can be said that adaptive ability means that the system can better deal with future uncertainty disturbances through active or passive learning. For the above three toughness characteristic ability relationships, the resistance and recovery phase after each disturbance provides learning opportunities for the adaptation phase, and the adapted urban transportation system can perform better in the resistance and recovery phases the next time it faces a similar shock of public health emergencies.

#### 2.1.2 Urban transportation system performance indicator

To comprehensively assess the toughness of the urban transportation system, based on the principles of comprehensiveness, objectivity, operability, and science, and taking into account the special characteristics of the urban transportation system in the face of the New Crown epidemic, the urban transportation infrastructure and the urban transportation passenger volume were finally selected as the research objects for constructing the system performance curve.

First of all, the urban transportation system is essential in urban economic development, livelihood improvement, normal operation, etc., and its infrastructure is one of the key foundations on which human society is highly dependent in the process of normal operation. In the face of the new crown epidemic, the proposed performance indicators of the urban transportation system should include the urban transportation infrastructure. Furthermore, according to the 36 central cities in China facing the disruption of the New Crown epidemic in 2020–2023, it is found that urban passenger traffic is the most affected. Therefore, this paper clarifies the connotation of urban transportation system toughness in the context of the New Crown epidemic, combines the characteristics of the study area and the degree of data accessibility, and constructs an urban transportation system performance indicator system with performance as the target layer and urban transportation infrastructure and urban passenger traffic as the indicator layer, which contains seven specific indicators, as shown in Table 1.

**Table 1:** Urban transportation system performance indicators.

Target layer	Indicator layer	Unit
Urban transportation system performance *Q*(*t*)	Urban road density *C*_1_	*km*/*km*^2^
	Public transport vehicle *C*_2_	*vehicles*
	Length of rail transit *C*_3_	*km*
	Cabs *C*_4_	*vehicles*
	Public tram traffic *C*_5_	10000*trips*
	Rail transit capacity *C*_6_	10000*trips*
	Cab traffic *C*_7_	10000*trips*

The parameters of the selected indicators about the urban transportation system are explained below:

Urban road density *C*_1_: the ratio of total road mileage to area in the built-up area of the central city. The road network density is the limitation of the development relationship between the length of the road and the area of the land, describing the road development level that should be in different city scales in terms of the length, but also has a great influence on the traffic control mode, the daily life of the residents and the transportation operation cost, and it is the basic guarantee for the supply of the urban transportation system.

Public transport vehicle *C*_2_: refers to the activities of providing basic travel services for the public in urban areas, utilizing public tram vehicles and their service facilities that meet the relevant standards, and operating in accordance with the approved routes, stops, times and fares. Urban public automobile and tram passenger transport is one of the most basic means of travel for the public, is an important part of urban public transportation, and is a universal service and people’s livelihood project that concerns the immediate interests of the public during the epidemic disruption.

Length of rail transit *C*_3_: Rail transit is a general term for fast, high-capacity public transportation powered by electricity and running on wheels and rails, and its length reflects the level of urban rail transit development. Urban rail transit can effectively relieve the traffic pressure of dense passenger flow within the city on a daily basis, even during epidemics.

Cabs *C*_4_: Taxi is an integral part of the comprehensive urban transport system, supplementing urban public transport and providing personalized transport services to the public. Because of their small carrying capacity and low contact between passengers, taxi trips were the first choice of most people traveling during the epidemic.

Public tram traffic *C*_5_, Rail transit capacity *C*_6_ and Cab traffic *C*_7_: refers to the actual number of passengers carried by the means of transportation of the above three modes of transport during the epidemic period. This indicator reflects the quantitative indicators of the services provided by the urban transportation system to the national economy and people’s life, and is also an important indicator for formulating and checking the production plan of urban transportation and studying the scale and speed of development.

#### 2.1.3 Entropy evaluation method

The entropy evaluation method is a method of objectively assigning weights to indicators based on the magnitude of their information entropy. In information theory, entropy is a measure of uncertainty information. The greater the degree of dispersion of an indicator, reflecting the large amount of valid information provided by the series, the greater its entropy value, which is manifested in a higher weight value; conversely, the smaller the degree of dispersion, the greater the entropy value and the lower the weight value. The entropy evaluation method can avoid the subjectivity bias of subjective assignment methods such as the hierarchical analysis method and expert scoring method and can avoid the lack of information caused by the principal component analysis method, so it is applied more in the comprehensive index evaluation system. The calculation steps of the entropy evaluation method are as follows:

(1) Construct the original matrix. Construct a matrix of *n*(cities)*m(indicators), noting that the value of the *j*th indicator for the *i*th city is *x*_*ij*_.

(2) Normalization of raw data. As the units of measurement of the various assessment indicators are not uniform, advanced data processing is required. Data normalization is used to calculate the weights of each level, as shown in Eq (1):

$$\begin{array}{c} x_{ij}^{\prime }=\frac{x_{ij}-min\left(x_{1j},\ldots ,x_{nj}\right)}{max\left(x_{1j},\ldots ,x_{nj}\right)-min\left(x_{1j},\ldots ,x_{nj}\right)} \end{array}$$ (1)

(3) Calculate the entropy value *e*_*j*_ for the *j*th indicator:

$$\begin{array}{c} P_{ij}=\frac{x_{ij}}{\sum_{i=1}^{n}x_{ij}} \end{array}$$ (2)

Where: *P*_*ij*_ is the numerical weight of the *j*th indicator for the ith city.

$$\begin{array}{c} e_{j}=-k\sum_{i=0}^{n}P_{ij}ln\left(P_{ij}\right) \end{array}$$ (3)

Where: *e*_*j*_ is the entropy value of the *j*th indicator, $k=\frac{1}{ln(n)}$, *e*_*j*_ ≥ 0.

(4) Calculate the information entropy redundancy:

$$\begin{array}{c} d_{j}=1-e_{j} \end{array}$$ (4)

Where: *d*_*j*_ is the variation index of the *j*th indicator.

(5) Calculate the weights of the indicators at each level:

$$\begin{array}{c} W_{j}=\frac{d_{j}}{\sum_{j=1}^{m}d_{j}} \end{array}$$ (5)

Where: *W*_*j*_ is the weight of the *j*th indicator.

#### 2.1.4 Urban transportation system performance calculation

The urban transportation system performance curve is mainly used to describe the state change of the urban transportation system when facing the new crown epidemic, which is a continuous function of time. Based on determining the weights of relevant indexes, combined with the index data at time t, the performance curve of the urban transportation system can be obtained through the calculation of Eq (6):

$$\begin{array}{c} Q(t)=\sum_{j=1}^{7}C_{j}^{\prime }\left(t\right)W_{j} \end{array}$$ (6)

where: *Q*(*t*) is the performance of the urban transportation system at moment *t*; $C_{j}^{\prime }\left(t\right)$ corresponds to the *j*th indicator normalized processing indicator at moment *t*; *W*_*j*_ is the weight corresponding to the *j*th indicator.

### 2.2 Quantitative calculation of urban transportation system toughness

This paper proposes the quantitative calculation of the toughness of urban transportation system as Eq(7) to Eq(10). When facing the new crown epidemic disturbance, the ratio of the cumulative performance of the urban transportation system to the cumulative performance of the system in normal operation is used to quantitatively calculate the system’s resistance, recovery, and adaptive ability. First, regarding the calculation of the resistance ability of the urban transportation system, the system performance is affected by the new crown epidemic at the moment of *t*_0_, and the system performance decreases at the moment of *t*_1_. Where the ratio of the area enclosed by the system’s performance *Q*(*t*) and the time axis to the area enclosed by the system’s performance *Q*_0_ and the time axis when it is not disturbed is used to characterize the system’s resistance ability:

$$\begin{array}{c} R_{1}=\frac{\int_{t_{0}}^{t_{1}}Q\left(t\right)dt}{\int_{t_{0}}^{t_{1}}Q_{0}dt} \end{array}$$ (7)

where: *R*_1_ is the resistance ability; *Q*_0_ is the system performance of the urban transportation system before the disturbance occurs; *t*_0_ is the time of disturbance occurrence; *t*_1_ The time at which the system performance decreases to a minimum value.

Secondly, about the recovery ability calculation of the urban transportation system. Facing the impact of the new crown epidemic disturbance, the performance of the system at the moment of *t*_1_ has increased to the moment of *t*_2_, where the ratio of the performance of the system *Q*(*t*) and the area surrounded by the time axis to the area surrounded by the disturbance down to the lowest performance of the system *Q*(*t*_1_) and the area surrounded by the time axis, is used to characterize the recovery ability of the system:

$$\begin{array}{c} R_{2}=\frac{\int_{t_{1}}^{t_{2}}Q\left(t\right)dt}{\int_{t_{1}}^{t_{2}}Q\left(t_{1}\right)dt} \end{array}$$ (8)

Where:*R*_2_ is recovery ability; *Q*(*t*_1_) is the performance of the urban transportation system at the moment of *t*_1_; *t*_2_ is the time for the system performance to recover to the maximum value.

Further, regarding the calculation of the adaptive ability of the urban transportation system. In the face of the new crown epidemic, after the government no longer carries out traffic control and other measures, the performance of the urban transportation system at the moment *t*_3_ naturally rebounds to the moment *t*_4_. Where the ratio of the area enclosed by the system’s performance *Q*(*t*) and the time axis to the area enclosed by the area enclosed by the lowest performance *Q*(*t*) and the time axis of the system that has been reduced to the system by the disturbance is used to characterize the system’s adaptive ability:

$$\begin{array}{c} R_{3}=\frac{\int_{t_{3}}^{t_{4}}Q\left(t\right)dt}{\int_{t_{3}}^{t_{4}}Q_{0}dt} \end{array}$$ (9)

Where: *R*_3_ is adaptive ability; *t*_3_ is the end time of the disturbance; *t*_4_ is the cutoff time of the study in this paper.

Finally, the comprehensive assessment of urban transportation system toughness is calculated as in Eq (10).

$$\begin{array}{c} R=\sum_{i=1}^{3}R_{i} \end{array}$$ (10)

Where: *R* is the urban transportation system toughness value; *R*_*i*_ stands for resistance ability, recovery ability, and adaptive ability.

## 3 Example analysis

### 3.1 Data collection

As shown in Table 2 below, from the aspects of urban GDP and urban resident population, it can be visualized that there are more obvious differences in the development of the four cities. Among them, Shanghai leads in terms of scale and degree of urban development, while Lanzhou is the last.

**Table 2:** Overview of urban development.

Sports event	Shanghai	Wuhan	Changchun	Lanzhou
City GDP/billion	38701	15616	6638	2887
Urban resident population/million	2488	1233	907	437
GDP per capita/yuan	155800	131441	77634	66680
Urban road area/ 10,000 square meters	31012	13517	7957	2838
Urban passenger traffic/million passengers	454108	141574	79882	93369
Number of infections/person	1505	68149	157	182
Hospitals and health centers/unit	398	362	229	116
Medical beds/beds	143638	91228	58936	282452
Tourism inflow/person	23605.71	25911.9	7223.48	482.14

Because of the actual impact of the new crown epidemic on the transportation system of major cities, and considering cities at different levels of development in China as the object of analysis, this paper selects four central cities, namely, Shanghai, Wuhan, Changchun, and Lanzhou, as examples. The relevant data for the case study are obtained from the China Urban Statistical Yearbook and the National Economic and Social Development Statistical Bulletin of each prefecture-level city. It should be clarified that the statistical data selected for this study are of city-wide caliber, but due to missing data, some of the indicators are replaced by the caliber of municipal districts, and the missing data of individual years are made up by the linear interpolation method. Among other things, data on urban transportation infrastructure are shown in Table 3. Among them, in terms of mean value: the mean value of public tram 9932.25, the mean value of rail transit length 355, the mean value of cab 22719.083; in terms of standard deviation: the standard deviation of public tram 5513.751, the standard deviation of rail transit length 317.521, the standard deviation of cab 9753.122. This shows that there is a difference in the cases of the selected cities, and it has the ability of comparability.

**Table 3:** Overview of urban transportation infrastructure.

Year—City	Public transport vehicle/*vehicles*	Length of rail transit/*km*	Cabs/*vehicles*	Urban road density/*km*/*km*^2^
2020-Shanghai	17668	729.21	37322	7.2
2021-Shanghai	17645	831	35317	7.21
2022-Shanghai	17300	831	34123	7.24
2020-Wuhan	11867	410	18078	6
2021-Wuhan	12030	484.2	18093	6.1
2022-Wuhan	11800	510.6	18188	6.1
2020-Changchun	6412	107.6	24432	5.5
2021-Changchun	6540	112.7	26386	5.6
2022-Changchun	6671	126.7	28496	5.6
2020-Lanzhou	3816	32	10766	6.42
2021-Lanzhou	3816	32	10640	6.56
2022-Lanzhou	3622	53	10788	6.71

### 3.2 Results of weighting calculations

Regarding the calculation of the weights of the performance indicators of the urban transportation system, universality and applicability should be achieved. The weights were calculated using the data of the 36 central cities in 2020, the time of the first outbreak of the new Crown Pneumonia epidemic, from the statistics of China’s Ministry of Transportation and Communications, and the results are shown in Table 4. It can be found that the indicator with the largest weight is the rail transportation capacity indicator, accounting for 27.988%, which is related to the large actual capacity of the rail transportation, and the indicator with the smallest weight is the urban road density indicator, which accounts for only 4.026%.

**Table 4:** The weighting of urban transportation system performance indicators.

Urban transportation system performance indicators	Information entropy value *e*	Information utility value *d*	Weight *W*_*j*_ (%)
Rail transit capacity/10000*trips*	0.764	0.236	27.988
Cabs/*vehicles*	0.825	0.175	20.652
Length of rail transit/*km*	0.863	0.137	16.211
Public transport vehicle/*vehicles*	0.905	0.095	11.244
Public tram traffic/10000*trips*	0.913	0.087	10.299
Cab traffic/10000*trips*	0.919	0.081	9.579
Urban road density/*km*/*km*^2^	0.966	0.034	4.026

### 3.3 Performance analysis of urban transportation systems

Before the disturbance of the new crown epidemic, the size of the initial performance of the urban transportation system in four cities, Shanghai, Wuhan, Changchun and Lanzhou, is shown in Table 5 below. Among them, the initial performance of Shanghai transportation system is 0.7924, ranking first, while the initial performance of Lanzhou transportation system is only 0.072, ranking last. This ranking is consistent with the actual development of the respective cities, which shows that the calculation of transportation system performance is practical and effective.

**Table 5:** Initial performance of urban transportation systems.

City	Initial performance	Ranking
Shanghai	0.7924	1
Wuhan	0.3024	2
Changchun	0.1865	3
Lanzhou	0.0720	4

Based on the above urban transportation system toughness assessment model, the performance results of four time-dependent urban transportation systems in Shanghai, Wuhan, Changchun, and Lanzhou were obtained by substituting the collected data into the calculation. The horizontal coordinates indicate the 39-month-long study period from January 2020 to March 2023, in months; the vertical coordinates indicate the performance level of the urban transportation system, in dimensionless values. In December 2022, China announced that there would be no more traffic control for the new crown epidemic, meaning that the government would no longer invest human and material resources in urban transportation interventions, and major cities would begin to enter a period of free adaptation.

#### 3.3.1 Shanghai transportation system performance

From Fig 2, it can be seen that the initial value of the performance of the Shanghai transportation system when it did not experience the new crown epidemic disturbance, *Q*_0_ = 0.79, is much higher than the initial value of the performance of the other three cities. It is intuitively obvious that the Shanghai transportation system experienced the larger scale of the three epidemic disturbances, and its transportation system functionality rapidly and significantly decreased. After the decline in the 2nd month, the system performance increases to a stable value at a decreasing rate over the next 5 months and exceeds the initial value of *Q*_0_ in the 7th month, and then experiences another small decline from the 12th to the 14th month, but quickly returns to a stable level in the following month. After reaching a peak of *Q*(*t*_22_) = 0.93 in the 22nd month, the system performance declines again, reaching an all-time minimum of *Q*(*t*_29_) = 0.49 in the 29th month. thereafter, it begins to recover and rise more sharply, recovering to a level slightly below the initial value of the performance value, *Q*_0_, in the 33rd month. finally, entering the acclimatization period, the system performance rises once again, until it reaches a level in the 39th month where it reaches a value of *Q*(*t*_39_) = 0.89, exceeding the initial value of performance *Q*_0_ = 0.79 when no new crown epidemic disturbance was experienced.

**Fig 2:** Shanghai transportation system performance curve.

#### 3.3.2 Wuhan transportation system performance

As shown in Fig 3, it is intuitively clear that the Wuhan transportation system experienced five new crown epidemic disturbances on a larger scale, and all of its transportation system functions declined significantly, with its system performance dropping to an all-time low of *Q*(*t*_2_) = 0.21 in the 2nd and 3rd months due to the impact of the city closure. the system’s performance value when it did not experience epidemic disturbances had an initial value of *Q*_0_ = 0.32. the system’s performance began to rise in the 3rd month onwards at a steady rate of increase, reaching *Q*(*t*_12_) = 0.36, which exceeds the initial value of performance *Q*_0_ at the 8th month. Immediately after, the system performance faces the impact of the epidemic from the 12th to the 14th month, and once again experiences a small decrease, but then quickly recovers to a stable level of around *Q*(*t*_15_) = 0.37 in the following month. In the 19th and 24th months, the system performance ebbs and flows again, with a similar degree of change compared to the previous change. After the 31st month, the system performance once again declines significantly at an even rate, and *Q*(*t*_35_) = 0.29. Finally, entering the adaptation period, the system performance once again rises to *Q*(*t*_39_) = 0.35 in the 39th month and reaches *Q*(*t*_37_) = 0.33 in the 37th month, exceeding the initial value of the system performance, *Q*_0_ = 0.32, when the system performance was not experiencing the disturbance of a new crown outbreak.

**Fig 3:** Wuhan transportation system performance curve.

#### 3.3.3 Changchun transportation system performance

As can be seen in Fig 4, the initial value of performance, *Q*_0_ = 0.19, was observed when the Changchun transportation system did not experience a new crown epidemic disturbance. The Changchun transportation system experienced three epidemic disturbances on a larger scale, and all of its transportation system functions declined. The system performance declined to a historical minimum of *Q*(*t*_2_) = 0.15 in the 2nd month, followed by a rapid increase to a stable value of *Q*(*t*_4_) = 0.17 in 2 months. the system performance exceeded the initial value of performance, *Q*_0_, in the 6th month, and slowly increased thereafter to the performance value of *Q*(*t*_25_) = 0.22 in the 25th month. in the 26th to 28th months, the system performance once again experiences a significant drop and takes 3 months to recover to a new peak level of *Q*(*t*_22_) = 0.23. Thereafter, in the 22nd month, the system performance drops once again to *Q*(*t*_36_) = 0.199 in the 36th month. finally, entering the adaptation period, the performance of the system starts to recover and rises considerably until it reaches *Q*(*t*_39_) = 0.23 in the 39th month, which is a significant increase in performance in comparison to the performance of the system in the period when the system did not experience the performance *Q*_0_ when the new crown epidemic was disrupted, a large improvement was obtained.

**Fig 4:** Changchun transportation system performance curve.

#### 3.3.4 Lanzhou transportation system performance

As shown in Fig 5, the initial value of the performance of the Lanzhou transportation system,*Q*_0_ = 0.07, is the lowest among the four cities when it does not experience the new crown epidemic disturbance. The performance of the Changchun transportation system dropped significantly seven times, and its performance curve is the most curved and variable. The system performance declined to the historical minimum of *Q*(*t*_2_) = 0.03 in the 2nd month, and declined to this extent in the 4th, 23rd, 35th, and 36th months, during which the system performance recovered near the initial value of the system performance in each case. It is not until the 36th month that the adaptation period is entered and system performance begins to resume a substantial increase because it is no longer under governmental control, reaching an all-time peak of *Q*(*t*_39_) = 0.084 in the 39th month, which is a performance improvement *Q*_0_ compared to the performance that would have been achieved had it not experienced the disruption of the new crown outbreak.

**Fig 5:** Lanzhou transportation system performance curve.

### 3.4 Toughness analysis of urban transportation systems

To deeply analyze the comprehensive toughness of the four urban transportation systems, based on the above system performance curves, combined with the proposed toughness calculation method, the comprehensive toughness and ranking of the transportation systems of each city are derived, as well as the magnitude of their resistance ability *R*_1_, resilience ability *R*_2_, and adaptive ability *R*_3_, and the results are shown in Table 6.

**Table 6:** Ranking the toughness of urban transportation systems.

City	*R*_1_	*R*_2_	*R*_3_	*R*	Ranking
Wuhan	4.81	5.23	1.03	11.07	1
Lanzhou	3.05	3.76	1.03	7.84	2
Changchun	2.82	1.18	1.18	7.37	3
Shanghai	2.67	2.99	0.98	6.64	4

In this new crown epidemic event, from the overall perspective of comprehensive toughness, Wuhan’s comprehensive transportation system toughness *R* = 11.07, far exceeds the toughness values of the other three cities’ transportation systems. Lanzhou, Changchun, and Shanghai come next in order, with little difference in system toughness. From the perspective of toughness characteristic ability, there are significant dissimilarities between the resistance and recovery ability of each city’s transportation system, but the adaptive ability does not differ much. The calculation of Eqs (7)–(9) shows that Wuhan has the highest comprehensive system toughness among the four cities because its resistance ability *R*_1_ = 4.81 and resilience ability *R*_2_ = 5.23 are the largest. Next, Lanzhou benefits from its resistance ability *R*_1_ = 3.05 and recovery ability *R*_2_ = 3.76, which is second only to Wuhan, and the combined down system toughness *R* = 7.84, which is in the second place. Further, Changchun’s adaptive ability *R*_3_ = 1.18, which is the largest among the four cities. Finally, Shanghai’s transportation system combined toughness *R* = 6.64, ranking last among the four cities.

### 3.5 Results and discussion

In the section of example analysis, the results are summarized as follows: first, in this paper, in terms of the weight of urban transportation system performance indicators, the weight of urban rail transportation capacity and the number of cabs is 27.988% and 20.652%, respectively, and its larger weight reflects the more obvious change of this indicator when disturbed by the epidemic; on the contrary, the weight of urban road density, which provides the basis of transportation supply, is only 4.026%, which reflects its smaller change when disturbed by the epidemic. On the contrary, the weight of urban road density, which provides the basis of transportation supply, is only 4.026%, reflecting that it changes less when disturbed by the epidemic. Secondly, in terms of urban transportation system performance, four cities with different levels of performance, namely Shanghai, Wuhan, Changchun and Lanzhou, are selected in the article, and the performance of the system fluctuates significantly under the influence of the epidemic in 39 months, with the biggest fluctuations coming from the second and third months of the epidemic. Finally, in terms of urban transportation system toughness, the size of resistance *R*_1_, resilience *R*_2_ and adaptation *R*_3_ of the four major cities were calculated to be different, and the size of the three capacities did not increase or decrease synchronously, resulting in Wuhan being ranked first in terms of urban transportation system toughness, which is in line with the actual situation during the epidemic in China.

In terms of discussion, this paper proves that the comprehensive assessment model of urban transportation system toughness based on urban transportation system toughness curves has practical significance and can provide reference for future urban toughness construction after example analysis. Further, the next research can also start from the toughness results, expanding the sample size of cities, choosing appropriate methods, exploring the reasons for the differences in the resistance *R*_1_, resilience *R*_2_, and adaptability *R*_3_ of transportation systems and toughness results of major cities, and arriving at the key influencing factors of toughness.

## 4 Conclusion

This paper establishes a comprehensive assessment model of urban transportation system toughness based on the urban transportation system function curve and proposes a calculation method to quantify the system toughness. In the context of the new crown epidemic event, the transportation system of four central cities in China is analyzed as an example, and the following conclusions are made.

- The entropy method is used to establish the performance curves of urban transportation systems, which can clearly describe the trend of the system performance over time during the whole cycle of the new crown epidemic. The performance of the transportation systems of the four cities shows a positive correlation with the level of development of the cities, and the ranking of the performance of the systems is Shanghai, Wuhan, Changchun, and Lanzhou in the order of the system performance. The transportation system performance of the four cities had different degrees of ups and downs and fluctuations due to the 39-month impact of the new crown epidemic, but all of them eventually recovered to a level of performance that exceeded the level of performance before the epidemic disturbance. Among them, Changchun recovered the most significantly and received a large performance improvement.
- Regarding the quantitative calculation of urban transportation system toughness, it is considered that the ability of the system to deal with the uncertainty disturbance is scientifically and intuitively reflected well in the three characteristic abilities of system toughness based on the urban transportation system performance curve through the change of the cumulative amount of system performance. That is, the three dimensions of resistance, recovery, and adaptive ability can be comprehensively and comprehensively quantitatively assessed for system toughness. Under the new crown epidemic event, the comprehensive urban transportation system assessment model established in this paper assesses the toughness of four different levels of urban transportation systems in China. The results show that Wuhan’s transportation system is at the maximum in terms of resistance and recovery ability, so its system toughness is the highest under the comprehensive assessment. In terms of adaptive capacity, there is not much difference among the four cities, mainly due to the time constraints of the study, which prevented the cities from fully demonstrating their adaptive capacity, which will only appear after the epidemic has ended or entered a period of normalization.

## Supporting information

S1 Data Supporting information file contains all the data for this manuscript. (ZIP)
